The article "Analysis of Clinical Effect after Treatment of Patients with Femoral Neck Fracture Using Total or Hemihip Arthroplasty" was retracted in 2022. Reason: concerns about the peer review.

# Analysis of Clinical Effect after Treatment of Patients with Femoral Neck Fracture Using Total or Hemihip Arthroplasty

**DOI:** 10.1155/2022/7422229

**Published:** 2022-02-22

**Authors:** Xin Zhao, Yongfeng Zhang, Ting Chen, Jianzhang Jia

**Affiliations:** ^1^No. 4 Department of Orthopaedics, Xianyang Central Hospital, Xianyang, Shaanxi, China; ^2^Orthopaedics Department, People's Hospital of Tongchuan, Tongchuan, China; ^3^Institute of Physical Education, Xizang Minzu University, Xianyang, Shaanxi, China

## Abstract

**Objective:**

To investigate the difference in clinical outcomes between total hip arthroplasty (THA) and hemiarthroplasty (HA) in patients with femoral neck fracture.

**Method:**

To retrospectively analyze 96 patients (96 hips) with femoral neck fracture treated in our hospital and distinguish them into THA group (50 patients with 50 hips) and HA group (46 patients with 46 hips) according to the difference of their chosen surgical procedure, and to compare the difference in perioperative indexes, postoperative hip function, occurrence of near and long-term complications, long-term imaging performance, and revision rate between the two groups.

**Result:**

The operating time, intraoperative blood loss, and total drainage were greater in the THA group than in the HA group (*P* < 0.05). At 6 months after surgery, the Harris score of the hip joint was higher in the HA group than in the THA group. At 3 years after surgery, the Harris score was higher in the THA group than in the HA group (*P* < 0.05). At 3 years after surgery, the excellent hip function rates were 86.00% and 67.39% in the THA and HA groups, respectively, with statistically significant difference between the groups. The incidence of long-term complications was significantly lower in the THA group than in the HA group (*P* < 0.05). The anteversion and abduction angles of patients in the HA group were smaller than those in the THA group at 6 months after surgery (*P* < 0.05). The WOMAC scores of the THA group were better than those of the HA group at 3 years after surgery (*P* < 0.05).

**Conclusion:**

Compared with hemiarthroplasty, total hip arthroplasty has a longer operative time and more postoperative bleeding, but the complication rate is relatively lower in the long term, and the patients have better long-term hip function recovery, so total hip arthroplasty is recommended for patients with femoral neck fracture with an expected survival time longer than 3 years.

## 1. Preface

The results of social research in recent years have shown [1] that the trend of aging in our society is gradually emerging and the prevalence of various degenerative diseases is increasing year by year. Clinical research has found [2] that the hip joint is an important ball and socket joint and plays an important role in maintaining the normal activities of the lower extremities, and data show [3] that the primary cause of mobility impairment in the elderly is hip fracture. One study predicted [4] that as the global population ages, the number of hip fracture will increase from the current 4.5 million to 21.3 million in 2050, with Asia accounting for about 45% of the total [5].

The article "Analysis of Clinical Effect after Treatment of Patients with Femoral Neck Fracture Using Total or Hemihip Arthroplasty" was retracted in 2022. Reason: concerns about the peer review.

Femoral neck fractures are more prevalent in orthopaedic clinics, accounting for around 3.59 percent of total body fractures, and are more common in older patients over 60. In recent years, the incidence of femoral neck fracture in senior persons in China has been growing year by year, and the total number of femoral neck fracture patients globally is predicted to reach 6 million by 2050 [6]. Hip arthroplasty is a typical therapeutic surgery for treating femoral neck fractures that may not only successfully relieve pain symptoms but also restore hip joint function as much as feasible, hence enhancing patients' quality of life [7]. Hip arthroplasty can be divided into total hip arthroplasty (THA) and hemiarthroplasty (HA), with THA requiring replacement of the femoral head and acetabulum and HA requiring replacement of the femoral head only. In recent years, there have been more clinical studies comparing the advantages and disadvantages of THA and HA [8, 9], but long-term follow-up of such patients has not been conducted. In this study, we propose to compare the effect of THA and HA on the near and long-term hip function of patients with femoral neck fracture, in order to provide a reference for choosing a more appropriate procedure for patients with femoral neck fracture.

## 2. Information and Method

### 2.1. General Information

A retrospective analysis of 96 patients (96 hips) with femoral neck fracture treated at our institution from April 2013 to April 2018 was performed, and they were distinguished into THA group (50 cases of 50 hips) and HA group (46 cases of 46 hips) according to the difference in their choice of procedure.

Inclusion criteria: (1) All patients were clearly diagnosed with femoral neck fracture, and single hip arthroplasty was performed. (2) All patients were conscious and able to cooperate with the study. (3) All patients had no previous hip surgery. (4) All patients had good hip interaction. (5) All patients had complete medical records.

Exclusion criteria: (1) Patients had combined active infection. (2) Patients had combined psychiatric disorders. (3) Patients had combined malignancy. (4) Patients had combined malignancy. (5) Patients had combined serious medical diseases. (6) Patients had combined coagulation dysfunction. (7) Patients had combined autoimmune system disorders. (8) Patients had long-term treatment with corticosteroids. (9) Patients had combined spinal disorders affecting lower limb movement. (9) Patients had combined pathological fracture or old fracture. (10) Patients had complicated primary diseases affecting hip function. (11) Patients had severe osteoporosis.

The article "Analysis of Clinical Effect after Treatment of Patients with Femoral Neck Fracture Using Total or Hemihip Arthroplasty" was retracted in 2022. Reason: concerns about the peer review.

Exclusion criteria: (1) Patients who missed the follow-up visit. (2) Patients who voluntarily requested to withdraw from the study.

### 2.2. Intervention Method

Routine blood tests, liver and kidney function, coagulation function, ECG, cardiac ultrasound, and chest DR were all conducted before surgery, and patients with complex diabetes and hypertension were given glucose and blood pressure medications. Patients with poor pulmonary function were given a combination of lumbar and stiff anesthesia, and the procedure was conducted in the contralateral position in both groups.

The THA group received biologic total hip arthroplasty, which entailed making an incision from the affected hip joint through the posterior approach of the greater trochanter to effectively expose the fracture, removing the femoral head, cleaning the acetabular glenoid labrum, cartilage, and femoral marrow, and finally implanting the biologic total hip joint. The surgical procedure was similar to that of the THA group, except that the femoral head was removed and the joint capsule was preserved before the bipolar femoral head was implanted. Both groups received postoperative drainage and antibiotics on a regular basis.

## 3. Observation Indicators and Evaluation Criteria

(1) Perioperative clinical indicators: the operating time, intraoperative blood loss, total drainage, and hospitalization time of the two groups were recorded, and the difference between the groups was compared. (2) Near and long-term hip function score: the hip Harris score was applied to assess the near and long-term hip function of the two groups, and this scale is commonly used to evaluate the effect of hip preservation and joint replacement, with a score out of 100, and a higher score means better function of the subject. (3) Excellent rate of near and long-term hip function: the excellent rate of the hip joint in the two groups was counted at 1 year, 2 years, and 3 years after surgery. And Harris score [10] of 90 or more was considered excellent, 80-89 was good, 70-79 was fair, and <70 was poor, and the excellent rate = (excellent + good)/total cases × 100%. (4) Incidence of near and long-term complications: the incidence of early complications (incision infection, dislocation, pulmonary infection, urinary tract infection, etc.) and long-term complications (hip pain, loosening, infection, acetabular wear, etc.) in the two groups were counted to carry out the intergroup difference comparison. (5) Postoperative imaging performance, the anteversion, and abduction angles of the hip joint at 6 months after surgery were recorded in the two groups and carried out the intergroup difference comparison. (6) Preoperative and postoperative WOMAC scale [11] scores. The WOMAC scale was used to assess the joint function of the patients at several time points before surgery, 6 months after surgery, 1 year after surgery, 2 years after surgery, and 3 years after surgery, respectively. A score of <80 indicates mild symptoms, 80-120 indicates moderate symptoms, and >120 indicates severe symptoms

The article "Analysis of Clinical Effect after Treatment of Patients with Femoral Neck Fracture Using Total or Hemihip Arthroplasty" was retracted in 2022. Reason: concerns about the peer review.

### 3.1. Statistical Method

SPSS22.0 statistical software was chosen to analyze the data collected in the study, where the measurement data were expressed as mean ± standard deviation; normal distribution and chi-square test were carried out—test was used for the difference between groups for data meeting normal distribution or chi-square. Mann-Whitney *U* test in a nonparametric test was applied for statistical inference for data with variance inconsistency, and the chi-square test was used for the difference between groups. The difference between groups was tested using the chi-square test, and the difference was considered statistically significant at *P* < 0.05. The GraphPad Prism 8.3 was used in this study [12].

## 4. Result

### 4.1. Comparison of Baseline Clinical Data between Two Groups of Patients

Gender, age, weight, disease diagnosis, anesthesia modality, Garden's staging, and replacement location were included in the baseline clinical data and used to compare the differences between the two groups. The results showed that none of the differences between the two groups in the above data were statistically significant (*P* > 0.05), implying that the two groups were comparable. See Table 1 for further information.

### 4.2. Comparison of the Difference in Perioperative Clinical Indicators between Two Groups of Patients

The operative time, intraoperative blood loss, total drainage, and hospital stay of patients in the THA and HA groups were included in the study, and an independent sample *t*-test was performed, which showed that the operative time, intraoperative blood loss, and total drainage of patients in the THA group were greater than those in the HA group, and the difference between the groups was statistically significant (*P* < 0.05). The difference between the two groups was not statistically significant (*P* > 0.05) when comparing the length of hospital stay. See Figure 1.

The article "Analysis of Clinical Effect after Treatment of Patients with Femoral Neck Fracture Using Total or Hemihip Arthroplasty" was retracted in 2022. Reason: concerns about the peer review.

### 4.3. Comparison of the Difference in Near and Long-Term Hip Function Scores between Two Groups of Patients

The hip Harris score was evaluated at 6 months, 1 year, 2 years, and 3 years postoperatively in both groups. The difference was statistically significant (*P* < 0.05) at 3 years postoperatively compared with 6 months postoperatively. At 6 months postoperatively, the Harris score in the HA group was higher than that in the THA group, and at 3 years postoperatively, the Harris score in the THA group was higher than that in the HA group (*P* < 0.05). See Figure 2.

### 4.4. Comparison of the Difference in the Rate of Excellent Long-Term Hip Function between Two Groups of Patients

The rates of excellent hip function at 1 year, 2 years, and 3 years postoperatively were evaluated by the Harris hip function score in both groups, and the difference between the groups was compared. The results showed that at 1 year and 2 years after surgery, the rates of excellent hip function in the THA and HA groups were 90.00% and 91.30%, 86.00%, and 82.61%, respectively, with no statistically significant difference between the groups (*P* > 0.05), while at 3 years after surgery, the rates of excellent hip function in the THA and HA groups were 86.00% and 67.39%, respectively. The difference between the groups was statistically significant (*P* < 0.05). See Tables 2–4.

### 4.5. Comparison of the Difference in the Incidence of Near and Long-Term Complications between Two Groups of Patients

The incidence of early complications (incisional infection, dislocation, pulmonary infection, urinary tract infection, etc.) in the two groups was counted, and the difference between the groups was compared, and the results showed that the difference between the two groups in terms of the incidence of early complications was not statistically significant (*P* > 0.05). The incidence of long-term complications (hip pain, loosening, infection, acetabular wear, etc.) in the two groups was counted and compared between the groups, and the results showed that the THA group had a significantly lower incidence of long-term complications than the HA group (*P* < 0.05). See Tables 5 and 6.

### 4.6. Comparison of Postoperative Imaging Performance between Two Groups of Patients

The results showed that the anteversion and abduction angles of patients in the HA group were smaller than those in the THA group, and the difference between the two groups was statistically significant (*P* < 0.05). The difference between the groups was statistically significant (*P* < 0.05), suggesting that the joint movement in the HA group was better than that in the THA group in the short term after surgery. See Figure 3.

The article "Analysis of Clinical Effect after Treatment of Patients with Femoral Neck Fracture Using Total or Hemihip Arthroplasty" was retracted in 2022. Reason: concerns about the peer review.

### 4.7. Comparison of Preoperative and Postoperative WOMAC Scale Scores between Two Groups of Patients

The WOMAC scale was used to assess the preoperative joint function of the two groups, and a comparison between the groups showed that the difference between the groups in the preoperative WOMAC scale dimensions was not statistically significant (*P* > 0.05), the HA group had lower pain, stiffness, and mobility scores than the THA group at 6 months postoperatively (*P* < 0.05), and the two groups had better WOMAC scores at 1 and 2 years postoperatively (*P* > 0.05). The difference between the WOMAC score groups for each dimension was not statistically significant (*P* > 0.05), and the THA group had better WOMAC scores than the HA group for each dimension at 3 years postoperatively (*P* < 0.05). See Figure 4.

## 5. Discussion

Femoral neck fractures are a form of fracture that often affects the elderly [13] and is a frequent orthopaedic ailment. The number of individuals with femoral neck fracture has risen in recent years as our population has aged and average life expectancy has increased [14]. According to the flow study, femoral neck fractures account for more than 53% of proximal femur fractures, with over half of the patients being old. Patients with femoral neck fractures are more likely to have fracture nonunion and femoral head necrosis as a result of events such as poor physical condition and a high incidence of underlying disorders, which may have a major influence on the patients' later lives. As a result, for individuals with surgical problems, vigorous surgical therapy is clinically suggested [15, 16].

The current clinical treatment measures for femoral neck fracture can be divided into three main categories: nonoperative treatment, internal fixation, and artificial hip replacement [17], among which nonoperative treatment is mainly applied to incomplete fracture or mild symptoms, and the applicable group is mostly young patients. However, elderly patients with femoral neck necrosis are limited by the less blood supply to the fracture site and difficulty in adapting to long-term bed rest. Data show that conservative treatment results in excellent outcomes of only 20%. Therefore, aggressive surgical interventions are mostly recommended in clinical practice [18]. Internal fixation is less intrusive, but it requires patients to be bedridden for a long period after surgery, and it has a poor postoperative healing effect on complicated and rotational fractures, increasing the likelihood of revision or crutches, which may have an influence on patients' quality of life [19]. Artificial arthroplasty is thus indicated for individuals who have a femoral neck fracture and are nevertheless physically capable of undergoing the treatment.

The article "Analysis of Clinical Effect after Treatment of Patients with Femoral Neck Fracture Using Total or Hemihip Arthroplasty" was retracted in 2022. Reason: concerns about the peer review.

In this research, we used a controlled group to assess the outcomes of two kinds of hip arthroplasty, THA and HA, on patients with femoral neck fracture. The findings indicated that the THA group had substantially greater operating time, intraoperative blood loss, and total drainage than the HA group, indicating that THA is more stressful and detrimental to patients than HA, as previous research [20] has shown. The results showed that at the 6-month postoperative time point, patients in the HA group had significantly higher hip Harris scores than those in the THA group, and there was no difference in the Harris scores at the 1-year and 2-year postoperative time points. At 3 years postoperatively, the Harris scores and good rates were significantly higher in the THA group than in the HA group. It has been pointed out that HA is less difficult, shorter, and less traumatic than THA, whereas THA requires acetabular replacement, resulting in a larger surgical incision and more complicated steps to separate the soft tissues, which is more traumatic to the patient's body and often results in poor recovery in the short term [21]. It was also pointed out that the factors affecting the recovery of patients after hip arthroplasty are complex, such as the surgical operation, the patient's body condition, and the preoperative anesthesia, which can affect the prognosis of patients [22, 23]. The analysis of this study concluded that the factors affecting the joint function of patients after hip arthroplasty are mainly the coordination of muscles, replacement prosthesis, and soft tissues. Although HA surgery is less traumatic and less painful for patients in the early postoperative period, however, over time, the coordination between the patient's femoral head and the acetabulum decreases, leading to complications such as acetabular wear and pain [23, 24], which is also reflected in the comparison of long-term postoperative complication rates between the two groups of patients in this study. In contrast, although patients undergoing THA had poor recovery of joint function in the short term due to surgical trauma, the results in this study showed that patients in the THA group had significantly better scores on both the Harris scale and the WOMAC scale at 3 years of follow-up. It has been noted that the pain level of patients after THA is significantly reduced and the quality of life is significantly improved, which may be related to the ability of THA to improve the accuracy of the pestle position of the acetabulum and femoral head through computer technology [25]. In this paper, the authors analyzed that compared with HA, THA can improve the degree of matching between the femoral head and the acetabulum, achieve a more precise union, and be closer to the biomechanics of the human lower limb, which helps patients achieve full weight bearing early after surgery and reduces the incidence of acetabular wear and prosthesis loosening, all of which have positive implications for improving the postoperative joint function of patients.

The article "Analysis of Clinical Effect after Treatment of Patients with Femoral Neck Fracture Using Total or Hemihip Arthroplasty" was retracted in 2022. Reason: concerns about the peer review.

In conclusion, compared with hemiarthroplasty, total hip arthroplasty has a longer operative time and more postoperative bleeding, but the complication rate is relatively lower in the long term and the patients have better long-term hip function recovery, so it is recommended that total hip arthroplasty be performed in patients with femoral neck fracture with an expected survival time of longer than 3 years. The limitations of this study are the small sample size and short follow-up time, which have a certain bias on the study results, and the conditions prevented further studies on the histology of cartilage wear and pseudomembrane properties of patients with both procedures, which are intended to be refined and revised in the follow-up.

## Figures and Tables

**Figure 1:** Comparison of the difference in perioperative clinical indicators between the two groups. Patients in the THA group had greater operative time (a), intraoperative blood loss (b), and total drainage (c) than the HA group, and the difference between the groups were all statistically significant (*P* < 0.05). The difference between the two groups was not statistically significant (*P* > 0.05) when comparing the length of hospital stay (d). # represents a statistically significant difference between groups comparing the same index.

**Figure 2:** Comparison of the difference in the near and long-term hip function scores between the two groups. Patients in the HA group had higher hip Harris scores than the THA group at 6 months postoperatively (*P*0.05), and at 3 years postoperatively, the THA group had higher Harris scores than the HA group (*P*0.05) (c), and at 3 years postoperatively, the THA group (a) and HA group (b) had similar hip Harris scores (b). When compared to the within-group pre-post comparison at 6 months postoperatively, the change in scores was statistically significant (*P*0.05). # denotes a statistically significant difference between groups when comparing the same metric.

**Figure 3:** Comparison of postoperative imaging performance between the two groups. The anteversion and abduction angles of patients in the HA group were smaller than those in the THA group, and the difference between the groups was statistically significant (*P* < 0.05). # represents a statistically significant difference between the groups comparing the same index.

The article "Analysis of Clinical Effect after Treatment of Patients with Femoral Neck Fracture Using Total or Hemihip Arthroplasty" was retracted in 2022. Reason: concerns about the peer review.

**Figure 4:** Comparison of preoperative and postoperative WOMAC scale scores between the two groups. The difference between the preoperative WOMAC scale scores for each dimension was not statistically significant (*P* > 0.05), the HA group had lower pain, stiffness, and mobility scores than the THA group at 6 months postoperatively (*P* < 0.05), the difference between the WOMAC scores for each dimension between the two groups at 1 and 2 years postoperatively was not statistically significant (*P* > 0.05), and the THA group had better WOMAC scores for each dimension than the HA group at 3 years postoperatively (*P* < 0.05). The difference between the WOMAC scores of the two groups at 1 and 2 years postoperatively was not statistically significant (*P* > 0.05), and the THA group had better WOMAC scores than the HA group in all dimensions at 3 years postoperatively (*P* < 0.05). # represents a statistically significant difference between groups comparing the same index.

**Table 1:** Comparison of the difference in general clinical data between the two groups ($\bar{x}\pm s$)/(*n* (%)).

General clinical information		THA group (*n* = 50)	HA group (*n* = 46)	*t*/*X*^2^	*P*
Gender	Male	28	24	0.141	0.707
	Female	22	22		
Average age (years)		55.19 ± 3.41	55.21 ± 3.51	0.034	0.973
Average weight (kg)		65.10 ± 5.98	65.08 ± 6.01	0.02	0.984
Disease diagnosis	Femoral head necrosis	21	18	0.123	0.718
	Hip osteoarthritis	17	18		
	Fracture of the neck of the femur	12	10		
Anesthesia method	Combined lumbar and rigid anesthesia	20	18	0.278	0.783
	Epidural anesthesia	13	12		
	Lumbar numbness	0	1		
	General anesthesia	17	15		
Garden typology	Type III	35	30	0.251	0.617
	Type IV	15	16		
Replacement position	Left side	24	22	0.0	0.986
	Right side	26	24		

**Table 2:** Comparison of excellent hip function rates between the two groups at 1-year follow-up (*n* (%)).

Group	Number of cases	Excellent	Good	Still acceptable	Poor	Excellent rate
THA	50	15 (30.00)	30 (60.00)	4 (8.00)	1 (2.00)	45 (90.00)
HA	46	16 (34.78)	26 (56.52)	3 (6.52)	1 (2.17)	42 (91.30)
*X* ^2^	—	—	—	—	—	0.048
*P*	—	—	—	—	—	0.827

**Table 3:** Comparison of excellent hip function rates between the two groups at 2 years of follow-up (*n* (%)).

Group	Number of cases	Excellent	Good	Still acceptable	Poor	Excellent rate
THA	50	14 (28.00)	29 (58.00)	6 (12.00)	1 (2.00)	43 (86.00)
HA	46	14 (30.43)	24 (52.17)	6 (13.04)	2 (4.35)	38 (82.61)
*X* ^2^	—	—	—	—	—	0.033
*P*	—	—	—	—	—	0.855

**Table 4:** Comparison of excellent hip function rates between the two groups at 3 years of follow-up (*n* (%)).

Group	Number of cases	Excellent	Good	Still acceptable	Poor	Excellent rate
THA	50	13 (28.00)	30 (60.00)	6 (12.00)	1 (2.00)	43 (86.00)
HA	46	11 (23.91)	20 (43.48)	10 (21.74)	5 (10.87)	31 (67.39)
*X* ^2^	—	—	—	—	—	4.697
*P*	—	—	—	—	—	0.03

The article "Analysis of Clinical Effect after Treatment of Patients with Femoral Neck Fracture Using Total or Hemihip Arthroplasty" was retracted in 2022. Reason: concerns about the peer review.

**Table 5:** Comparison of the incidence of early postoperative complications between the two groups (*n* (%)).

Group	Number of cases	Incision infection	Dislocation	Lung infection	Urinary tract infection	Total incidence
THA	50	0 (0.00)	3 (6.00)	1 (2.00)	1 (2.00)	5 (10.00)
HA	46	0	2 (4.35)	1 (2.17)	1 (2.17)	4 (8.70)
*X* ^2^	—	—	—	—	—	0.048
*P*	—	—	—	—	—	0.827

**Table 6:** Comparison of the incidence of late postoperative complications between the two groups (*n* (%)).

Group	Number of cases	Hip pain	Loosen up	Infection	Acetabular wear	Total incidence
THA	50	3 (6.00)	0 (0.00)	1 (2.00)	0 (0.00)	4 (8.00)
HA	46	7 (15.22)	2 (4.35)	2 (4.35)	0 (0.00)	11 (23.91)
*X* ^2^	—	—	—	—	—	4.602
*P*	—	—	—	—	—	0.032

## Data Availability

The data used to support the findings of this study are included within the article.
